# Cross-Sectional Analysis of Impulse Indicator Saturation Method for Outlier Detection Estimated via Regularization Techniques with Application of COVID-19 Data

**DOI:** 10.1155/2022/2588534

**Published:** 2022-05-06

**Authors:** Sara Muhammadullah, Amena Urooj, Muhammad Hashim Mengal, Shahzad Ali Khan, Fereshteh Khalaj

**Affiliations:** ^1^Department of Economics and Econometrics, Pakistan Institute of Development Economics, Islamabad, Pakistan; ^2^World Health Organization, Pakistan; ^3^Vice-Chancellor of Health Services Academy Islamabad, Pakistan; ^4^Department of Mathematics and Statistics, Parand and Robat Karim Branch, Islamic Azad University, Tehran, Iran

## Abstract

Impulse indicator saturation is a popular method for outlier detection in time series modeling, which outperforms the least trimmed squares (LTS), M-estimator, and MM-estimator. However, using the IIS method for outlier detection in cross-sectional analysis has remained unexplored. In this paper, we probe the feasibility of the IIS method for cross-sectional data. Meanwhile, we are interested in forecasting performance and covariate selection in the presence of outliers. IIS method uses Autometrics techniques to estimate the covariates and outlier as the number of covariates *P* > *n* observations. Besides Autometrics, regularization techniques are a well-known method for covariate selection and forecasting in high-dimensional analysis. However, the efficiency of regularization techniques for the IIS method has remained unexplored. For this purpose, we explore the efficiency of regularization techniques for out-of-sample forecast in the presence of outliers with 6 and 4 standard deviations (SD) and orthogonal covariates. The simulation results indicate that SCAD and MCP outperform in forecasting and covariate selection with 4 SD (20% and 5% outliers) compared to Autometrics. However, LASSO and AdaLASSO select more covariates than SCAD and MCP and possess higher RMSE. Overall, regularization techniques possess the least RMSE than Autometrics, as Autometrics possesses the least average gauge at the cost of the least average potency. We use COVID-19 cross-sectional data collected from 1 July 2021 to 30 September 2021 for real data analysis. The SCAD and MCP select CRP level, gender, and other comorbidities as an important predictor of hospital stay with the least out-of-sample RMSE of 7.45 and 7.50, respectively.

## 1. Introduction

The ordinary least squares (OLS) approach has been a widely chosen technique among the numerous available methods in regression analysis because it is computationally straightforward and possesses the best linear unbiased estimate. However, it possesses strong assumptions on the distribution of error (*ε*) termed as *ε* ~ *N* (0, *σ*), which is usually violated while dealing with real data analysis. The leading cause of distortion is outliers, which violates the normality assumption of residuals. Outlying data in the dependent and regressor variables pose a risk to least squares regression since they might negatively impact the estimate if they go unreported. Even cross-sectional data with high quality contain outliers; however, it is rare in time series economic data (because of the differencing variables) [1].

Robust regression techniques are used significantly in the literature of outlier presences. Langford and Lewis [2] well defined an outlier as data points that look inconsistent with the rest of the data. Such influential points are frequently concealed from the user since they do not always appear in the standard least-squares residual graph [3]. Zaman et al. [1] indicate that the OLS residuals are ineffective in finding outliers in small and big sample sizes, whereas Rousseeuw and Leroy [4] demonstrate several real data sets in which the OLS residuals miss to detect any outliers despite significant outliers. However, new statistical procedures have been proposed that are less susceptible to outliers; Rousseeuw [5] introduced the primary feasible robust regression estimators (least median squares (LMS), least trimmed squares (LTS), and variations) that perform correctly even when a high number of outliers are present. Huber M estimation, MM estimation, least absolute value method (LAV), and S estimation are examples of robust approaches [6–8]. A conspicuous technique is established on Huber's M-estimators, which offer robustness in location parameters. Regrettably, generalizations to regression models miss the mark to accomplish robustness. As Rousseeuw [5] illustrates, regression M-estimators likewise have a 0% breakdown value. The generalization of MM-estimators likewise fails to attain large breakdown values. A direct method to robust regression is to use LTS analysis in huge residuals. The LTS analysis discards outlying observations and then can run a standard OLS regression, proposed in Rousseeuw [5]. However, removing too many data points in the case of too many outlier observations turns the risk of the final regression model not reflecting the association that the econometrician wants to assess [1].

On the contrary, Doornik [9] and Johansen and Nielsen [10] illustrate the impulse indicator saturation (IIS) as a robust estimator. Similarly, Johansen and Nielsen [10] describe and demonstrate that a split-sample estimator for the indicator-saturated regression model is a one-step M-estimator that is iterated twice. Doornik [9] illustrates that robustified least squares and indicator saturation are more efficient than least trimmed squares. When the covariates are static and only outliers occur in the dependent variable's data, M estimation works effectively. The impulse indicator saturation method was initially designed to detect unidentified numbers of outliers with indefinite magnitudes at uncertain points in the sample, together with the start and end of observations [11]. However, the step indicator saturation (SIS) method is a modified version of IIS techniques for multiple break detection. Indicator saturation (IS) is used as a border term that detects outlier (via IIS) and multiple break shifts (via SIS) and simultaneously estimates the underlying modeling [9–13].

As the IS method possesses the number of candidates regressor more than the number of data points, the OLS estimates fail to estimate the thriving model. However, Autometrics handles such phenomena efficiently regardless of candidate regressors exceeding the number of observations; due to this reason, IS method is feasible to estimate via Autometrics. Autometrics uses extending and contracting multiple-path search algorithms with user-specified significance levels through the model selection process. However, the choice of the significance level is the trade-off between the irrelevant and relevant dummy indicators or regressors, with tight significance level (0.001) significant variable omitted in the final model whereas, with 0.05 significance level, the model consists of irrelevant regressors [13–15].

Other than Autometrics, regularization techniques are emerging techniques when the number of covariates excel the number of data points (observations); some of these popular techniques are Least Absolute Subset Selection Operator (LASSO), Adaptive LASSO, Smoothly Clipped Absolute Deviations (SCAD), and Minimax Concave Penalty (MCP) [16–19]. However, every few studies compare the computational efficiencies of Autometrics with regularization techniques [20] [21–23] for covariate selection and forecasting under the normality assumption. They do not consider outliers with the IIS setup. As it is challenging to choose the level of significance for thriving models in Autometrics, the regularization techniques can be used as an alternative model selection method in this case. Up to date, the prevailing studies do not compare the computational efficiency of regularization techniques with Autometrics in cross-sectional analysis with outlier in IIS setup. This study is aimed at analyzing the computational efficiency of regularization techniques with IIS setup in cross-sectional phenomena. The computational proficiency of these methods is evaluated with potency, gauge, and out-of-sample Root Mean Square Error (RMSE) in the simulation experiment. For the simulation experiment, the Data Generating Process (DGP), we opt with the orthogonal regressors and possess three scenarios 5%, 10%, and 20% outlying observations with 4 and 6 standard deviation (SD). Meanwhile, in DGP, we intake orthogonal cases for this purpose we use some well-known orthogonal techniques of regularization like LASSO, Adaptive LASSO, Smoothly Clipped Absolute Deviation (SCAD), and Minimax Concave Penalty (MCP) [16–19].

Outlier detection is a rapidly developing procedure in the healthcare and medical data industries, and it is a significant source of concern. Hauskrecht et al. [24] study data-driven outlier-based surveillance and forewarning system that uses data from former patient cases. Wilson et al. [25] used the outlier identification method for hypoglycemia safety in patients, calculating a flair outlier value within a year, comparator group, and A1c threshold while considering at hazard population proportions. Jyothi et al. [26] used outlier detection in healthcare data, a key source of concern for health insurers. The development of a Supervised Outlier Detection Approach in Healthcare Claims (SODAC) and carried out in two parts. Noma et al. [27] offer optimal effect measures for network meta-analysis models with mislaid outcomes and appropriate degree of freedom adjustments. The real data application of the IIS method in healthcare and medicine with outliers for cross-sectional analysis does not exist in the current literature [24–30]. To probe the efficacy of the IIS method estimated via regularization techniques for real data techniques, we use COVID-19 cross-sectional surveillance data, which has been collected from July 2021 to 30 September 2021 in Isolation Hospital and Infectious Treatment Center (IHITC) Islamabad. We aim to analyze the factors associated with prolonging the length of hospital stay of COVID-19 patients in the capital territory of Islamabad.

## 2. Outlier Detection and Model Selection Techniques

### 2.1. Impulse Indicator Saturation

Impulse indicator saturation is a popular method of outlier detection as it already dominates the existing outlier selection techniques like least trimmed squares (LTS), M-estimator, and MM-estimator [9, 10]. Usually, in multivariate regression, we assume that error is normally distributed, which is usually violated in real data analysis. In the equation below, we assume that error is not normally distrusted, and *α* is the intercept of the model, *y* is the continuous dependent variable, and *x*_*ji*_ is the orthogonal regressors, where *j* = 1, 2, 3, ⋯, *k* number of orthogonal regressors and *i* = 1, 2, 3, ⋯, *n* observations.

(1) $$\begin{array}{c} y_{i}=\alpha +\overset{k}{\underset{j=1}{\sum }}\beta_{j}x_{ji}+\varepsilon_{i}. \end{array}$$

As in equation (1), the error is not normally distributed due to the presence of an outlier; in this case, the IIS method introduces an impulse dummy indicator to each of the data points, and the above equation would be

(2) $$\begin{array}{c} y_{i}=\alpha +\overset{k}{\underset{j=1}{\sum }}\beta_{j}x_{ji}+\overset{n}{\underset{i=1}{\sum }}\gamma_{i}I+\varepsilon_{i}, \end{array}$$

where

(3) $$\begin{array}{c} I=\left[\begin{array}{ccccc} 1 & 0 & 0 & \cdots & 0\\ 0 & 1 & 0 & \cdots & 0\\ 0 & 0 & 1 & \ddots & 0\\ \vdots & \vdots & \vdots & 1 & \vdots \\ 0 & 0 & 0 & 0 & 1 \end{array}\right]. \end{array}$$

Here, *I* is an identity matrix of each corresponding observation in the above equation. *I*_1_′ = (1, 0, 0, ⋯⋯.., 0), *I*_2_′ = (0, 1, 0, 0, ⋯⋯, 0), and *I*_*i*_′ = (0, 0, 0, ⋯⋯., 1). The OLS estimate is not feasible to estimate the above Generalized Unrestricted Model (GUM). Estimating the above equation is possible because Autometrics (created on general-to-specific modeling) is used to detect the outlier and estimate the model instantaneously. In the general-to-specific methodology, each observation would have one dummy variable, and additional exogenous variables can be considered that possibly distress the dependent variable [10, 12].

### 2.2. Model Selection Methods

There are two main fields of model selection methods when covariates are higher than the number of data points: the regularization technique and the classical (general-to-specific, Autometrics) approach. The classical method (Autometrics) is initiated by a saturated model and uses the multipath search process to eliminate insignificant covariates. The model selection is primarily dependent on the preset significance threshold. On the other hand, the regularization approach applies sparsity to the *p*-dimensional vector of parameters, resulting in numerous parameters of covariates equal to zero. This approach resolves the issues that arise in high dimensionality. We go through each of these methods further; however, we only looked at orthogonal regularization approaches.

#### 2.2.1. Autometrics

The general-to-specific model procedure, presented by Hoover et al. [31], combines several components of Krolzig and Hendry [32]. PcGets is a second-generation extension of general-to-specific method; it extends and clarifies Hoover and Perez's methodology [32, 33]. Modifying the existing techniques, Doornik [9] introduced Autometrics which is based on the same concept of general to specialized (gets) modeling. Autometrics is a third-generation algorithm based on the same concept of PcGets.

Autometrics employs a tree path search that includes multistep simplifications along several pathways. The GUM contains all covariates at first and estimates them using the OLS technique, removing statistically insignificant covariates; the compact model's reliability is tested at each individual stage to guarantee consistency with the test diagnostics. Autometrics employs a tree-path exploration strategy that involves multiple multistep simplifications. The ultimate models are constructed that used a tree-path approach and assessed using screening procedures; the parameters are automatically eliminated if the parameter estimates are statistically irrelevant. Autometrics retests their union once a high number of terminal models are discovered. A novel GUM is formed once the “surviving” terminal models are merged, permitting another tree-path search repetition. The whole search procedure is completed by reexamining the terminal models and their consolidations. If a large number of models pass all of the tests, the final decision is made on specified information criteria.

The test diagnostics are being used to ensure the simple models, whereas inclusive tests are used to resolve several terminal models. Epprecht et al. [20] argue that Autometrics is a kind of black box technique. While developing modeling techniques, the user can select among 1-cut and tight significance level and nominal significance level. The multipath technique in Autometrics identifies multiple breaks/outliers more effectively and has reduced estimator variance [34]. The multipath technique eliminates path reliance by employing a tree structure and alike stepwise sequential backward, an integral function of the gets package in R software [15].

#### 2.2.2. Regularization Techniques

Other than Autometrics, regularization approaches manage saturated models with irrelevant variables even if the amount of regressors excel the quantity of data points (observations), shrinking the irrelevant parameters to zero with a nearly biased estimate. The Least Absolute Shrinkage and Selection Operator (LASSO) was introduced by Tibshirani [17]. It is a standard estimation method in a linear regression framework due to its decreased computing cost. The LASSO does not hold an oracle property; Zou [19] proposed Adaptive LASSO. The regularization penalty is defined in

(4) $$\begin{array}{c} {\hat{\gamma }}_{j}=\text{argmi}{\text{n}}_{\hat{\gamma }}\overset{n}{\underset{i=1}{\sum }}\left(y_{i}-\alpha -\overset{k}{\underset{j=1}{\sum }}\beta_{j}x_{ji}-\gamma_{i}I\right)+\lambda p\left(\left|\gamma_{j}\right|\right). \end{array}$$

In the above equation, *y* is a continuous dependent variable, *x* is an orthogonal covariate, and *I* is the impulse dummy for outliers. The following regularization techniques contemplate different choices for the penalty function, which is summarized in Table 1.

(5) $$\begin{array}{c} \left(\text{Lasso}\right)p_{\lambda_{j}}\left(\left|\gamma_{j}\right|\right)=\lambda_{j}\left|\gamma \right|. \end{array}$$

The “*L*1 penalty” for the LASSO estimator is the subsequent term in the preceding equation, and it primes to a sparse solution with a very precise set of parameters exactly equivalent to zero through a particular level of bias. The choice of *λ* determines the quantity of reduction, and it varies from 0 < *λ* < ∞.

Zou [19] revealed that the LASSO method violated the oracle property and proposed the Adaptive LASSO as a modest and effective alternative. On the other hand, the coefficients in LASSO are altogether penalized similarly in the “*L*1 penalty.” Nevertheless, in the AdaLASSO method, individual parameter is assigned its own weight. Zou [19] demonstrated that if the weights are data-dependent and correctly set, the AdaLASSO may have the best outcomes and exhibit the oracle property.

(6) $$\begin{array}{c} \left(\text{Adaptive Lasso}\right)\;p_{\lambda_{j}}\left(\left|\gamma_{j}\right|\right)=\lambda_{j}w_{j}\left|\gamma \right|,\;\text{where }w_{j}={\left|{\overset{\wedge }{\gamma }}_{j}\right|}^{-\tau }. \end{array}$$

${\hat{w}}_{j}=1/{\left|{\hat{\gamma }}_{j}^{*}\right|}^{\tau }$ , *τ* > 0, and ${\hat{\gamma }}_{j}^{*}$ is a preliminary parameter estimate. The weights of irrelevant parameters approach infinity as the sample increases, whereas relevant parameters approach a finite constant. Zou [19] suggested using the OLS technique to estimate ${\hat{\gamma }}_{j}^{*}$. On the other hand, the OLS approach does not work as soon as the amount of candidate regressors excel the quantity of data points (observations). A ridge estimate might be used as a preliminary estimator in this scenario.

Fan and Li [16] introduced a new approach that satisfied the condition of unbiased, sparsity, and continuity known as Smoothly Clipped Absolute Deviation (SCAD).

(7) $$\begin{array}{c} \text{SCAD}=\lambda \left\{\begin{array}{c} \left|\gamma \right|\text{ if }\left|\gamma \right|\leq \lambda ,\\ -\frac{\left(\gamma^{2}-2a\lambda \left|\gamma \right|+\lambda^{2}\right)}{2\left(a+1\right)\lambda }\text{ if }\lambda <\left|\gamma \right|\leq a\lambda \text{ and}\\ \frac{1}{2}\left(a+1\right)\lambda \text{ if }\left|\gamma \right|\geq a\lambda \end{array}\right\}. \end{array}$$

Distinct to LASSO, SCAD uses two tuning parameters *α* and *λ*; *P*(*γ* | *λ*, *α*) of SCAD method is known as folded concave penalty that depends on *λ* in a nonmultiplicative way; hence, *λP*(*α*) = *P*(*α* | *λ*). In addition, the tuning parameter (*λ*) affects the penalty's concavity. The objective function's intensification is determined by *λ* and *α*, *λ* being chosen via cross-validation and *α* is fixed equal to 3.7 [16].

Zhang [18] proposed the Minimax Concave Penalty (MCP), a nonconvex regularization approach that uses spares zone up to a specified choice of threshold to produce an unbiased estimate.

(8) $$\begin{array}{c} \text{MCP}=\lambda \left\{\begin{array}{c} \left(\lambda -\frac{\left|\gamma \right|}{\alpha }\;\mathrm{sign}\left(\gamma \right)\text{ if }\left|\gamma \right|\leq \alpha \lambda \right.\\ 0\text{ if }\left|\gamma \right|>\alpha \lambda \end{array}\right\}. \end{array}$$

MCP employs the *p*_*j*_(|*γ*_*j*_|; *λ*; *α*) regularization pathway, which is constructed on a family of nonconvex penalty functions through two tuning parameters *λ* and *α*, whereas *α* is constant and *λ* is chosen by cross-validation. The *λ* tuning parameter regulates the degree of penalty shrinking and concavity. Because the maximum concavity is minimized, MCP minimizes the convexity of the spares to a greater extent [18]. SCAD and MCP estimates fall to the folded concave penalty family since the *P*() penalty function is neither convex nor concave.

#### 2.2.3. Selection Criteria for Tuning Parameter

The selection of tuning parameter is critical since it determines the complication of the chosen model. The selection of the suitable tuning parameters results in a compact model with accurate forecast performance. In order to achieve prediction optimality, the tuning parameter is commonly selected by a cross-validation technique. The aim is to retrieve the primary collection of sparse covariates. Covariate selection typically needs a more substantial penalty parameter than optimum prediction [35]. The information criteria like Akaike Information Criteria (AIC) or Bayesian Information Criteria (BIC) are used as another approach for penalizing the likelihood through the degrees of freedom of the fitted model. Degrees of freedom are frequently used to measure the complication of a model fit, and we can use them to decide how much regularization to utilize. Meanwhile, in terms of covariate selection and out-of-sample forecast, WLAdaLASSO with a BIC-based tuning parameter possesses optimal results [23, 36].

(9) $$\begin{array}{c} \text{BIC}=n\log\left({\overset{\wedge }{\sigma }}^{2}\right)+\log\left(n\right)+df\hat{\left(y\right)}, \end{array}$$

whereas ${\overset{\wedge }{\sigma }}^{2}=n^{-1}\sum_{i=1}^{n}{\left(y_{i}-{\overset{\wedge }{y}}_{i}\right)}^{2}$ and $df\hat{\left(y\right)}$ signifies the degrees of freedom of the fitted model. The BIC-based tuning parameter, on the other hand, is superior to cross-validation for covariate selection, although there is no theoretical justification [35]. Henceforth, the BIC-based tuning parameter is used for outlier and covariate selection in simulation and real data analysis.

### 2.3. Theoretical Assessment

The study is aimed at evaluating the out-of-sample forecasting performance of regularization methods in the presence of an outlier in the IIS setup. However, other than out-of-sample RMSE, we also emphasize the average gauge and potency in the simulation study. Gauge is defined as the empirical null retention frequency of how insignificant variables/outliers are reserved, whereas potency is identified as correct covariate/outlier identifications. The assessment of regularization methods and Automatics was evaluated via an accurate zero identification taken as potency and improper zero identification denoted as gauge [37]. If the considered techniques appropriately classify the model, the evaluations of the subsequent parameters should be expected:

1. The gauge is getting close to the significance level (0.05) or the tight significance level (0.01 or 0.001)

(10) $$\begin{array}{c} E\left(\frac{\hat{k_{\text{irr}}}}{k_{\text{irr}}}\right)⟶\alpha . \end{array}$$

(2) When estimating techniques are used to estimate the exact model efficiently, potency approaches 1

(11) $$\begin{array}{c} E\left(\frac{\hat{k_{\text{rel}}}}{k_{\text{rel}}}\right)⟶1. \end{array}$$

For out-of-sample RMSE, we randomly trained our model on 90% of observations, and 10% of observations were discarded to test the model's accuracy in terms of RMSE [23]. The RMSE of regularization techniques, even in an outlier, is expected to be smaller than Autometrics. However, LASSO will retain more regressor variables than SCAD, MCP, and Autometrics.

## 3. Data Generating Process and Simulation Experiment Result

The Data Generating Process (DG) in this section has opted from [9] where the models consist of irrelevant regressors and outliers. We assumed well scatter outlier among DGP with 5%, 10%, and 20% observations, which is different from Doornik [9], as it has been illustrated 20% outlier at the end of observations with magnitude coefficients equal to 6 in the static DGP, where the DGP can be defined as

(12) $$\begin{array}{c} y_{i}=0.1+\overset{k}{\underset{j=1}{\sum }}\beta_{j}x_{ji}+6\left(\tau \right)+\varepsilon_{i}, \end{array}$$

where *β*_1_ = ⋯⋯ = *β*_*k*∗_ = 1 whereas *k*^∗^ is equal to 10 and the rest of the other beta coefficients equal zero, and *k* = 20 with *i* = 1, 2, ⋯, 100 observations. The regressors *x*_*ji*_ ~ IID(0, 1) and *ε* ~ IID(0, 1), whereas the outlying observations (*τ*) are equal to 5%, 10%, and 20% with 6 SD and 4 SD of error term. To estimate the above DGP, we use the Generalized Unrestricted Model (GUM) and introduce an impulse dummy indicator for each observation in the model. The experiment is repeated 1000 times.

### 3.1. Simulation Experiment Result

The comparison is assessed under scenarios with 5%, 10%, and 20% scattered outliers with 6 SD and 4 SD. The glmnet package for R software is used to estimate LASSO and AdaLASSO. For MCP and SCAD estimation, we use the ncvreg package of R; the ncvreg package uses a coordinate descent algorithm, while for Autometrics we use the gets package of R. To achieve our study objective, we use a static DGP with orthogonal covariates and dummy indicator saturation opts from Doornik [9]. It provides a convenient base for comparing regularization techniques with Autometrics in the presences of outliers. Outcomes of the simulated scenarios are obtainable in Table 2. Table 2 illustrates the average gauge and potency Autometrics and regularization techniques; however, the RMSE error of the out-of-sample forecast has been presented below. We use Auto as an acronym of Autometrics in the tables and figures, and the computational efficiency of Autometrics is assessed with 0.05 and 0.01 significance levels.

Table 2 demonstrates the results of regularization techniques with Autometrics for covariate selection and outlier detection in potency and gauge. The result indicates that with a 20% and 6 SD outlier, Autometrics performs worse in average potency among all existing techniques. On the contrary, LASSO possesses the highest gauge and potency among regularization techniques. Meanwhile, SCAD and MCP accomplish similar performance in both average gauge and potency. The simulation result specifies that as the outlier percentage decreases to 10%, the performance of considered methods increases in average potency. However, the performance of SCAD and MCP improved with both gauge and potency. With 5% outlying observation, the considered techniques improved further. The SCAD and MCP estimate retains 60% average potency with an average gauge equal 5%.

In Table 3, the result indicates that with 20% and 4 SD outliers, Autometrics performs worse among all existing techniques in average potency; however, the average potency of SCAD and MCP drastically increased compared to outliers with 6 SD. Meanwhile, significant improvement in the average potency of the regularization technique with 4 SD outlier has been observed over 6 SD, whereas the performance of the average gauge remains the same in both seniors. On the contrary, LASSO possesses the highest gauge and potency among regularization techniques, similar to outliers with 6 SD. Compared to LASSO and SCAD, MCP performs significantly in gauge equal to 0.095 and 0.114 of SCAD with a 5% outlier. The simulation result shows that as the outlier percentage decreases to 10%, the performance of considered regularization methods decreases in average potency, whereas the average gauge remains similar to 20% outliers.

Overall, the simulation result indicates that outliers with 4 SD and 5% outlying observation regularization techniques perform better than 6 SD outliers in terms of average potency, whereas the average gauge of regularization techniques with 6 SD is lower than 4 SD outliers. The Autometrics possesses the least average gauge in all scenarios (5%, 10%, and 20%, 6 SD and 4 SD) at the rate of the smallest average potency among all considered techniques. In contrast, LASSO possesses the highest potency and gauge of all other methods.

Figures 1–3 represent the out-of-sample forecasting performance of the considered methods. The graphs illustrate that the average RMSE error of LASSO with 20% and 10% outlier observations is the least among all considered techniques. The result aligns with existing literature as LASSO possesses the least forecasting error and selects a more irrelevant regressor (which can be observed from Table 1) [38]. However, with less than 5% outlier observations, the SCAD and MCP possess the least RMSE 3.03 than all other techniques, even less than Autometrics. We observed that Autometrics with 5% outliers possesses the least gauge but retain higher RMSE than SCAD and MCP. Autometrics with 0.05 level of significance possesses the least RMSE than 0.01 level of significance, the fact that Autometrics with 0.01 level of significance omits relevant regressors which increases the average RMSE.

There is a significant improvement in average RMSE with 4 SD with 5% and 20% outliers compared to 6 SD with 5% and 20% outliers. This difference can be justified as with 5% and 4 SD outliers, the average potency is higher (means that method correctly identified the correct variables/dummy indicator) compared to 6 SD, which ultimately impact the out-of-sample RMSE, and the same pattern can be observed with 20% outliers and 6 SD the average potency is least due to this reason the out-of-sample RMSE increases. However, the average potency of 20% outliers with 4 SD is close to 1 for regularization techniques; due to this, the out-of-sample RMSE of regularization techniques is the least compared to 6 SD, as shown in Figure 3. On the contrary, as 10% and 4 SD and 10% and 6 SD outliers, the performance of considered methods is aligned in average potency, and consequently, the average RMSE are almost similar observed in Figure 2.

## 4. Real Data Analysis

Coronavirus disease 2019 (COVID-19) is a global outbreak triggered by coronavirus 2, which origins severe acute respiratory illness (SARS-CoV-2). The World Health Organization declared COVID-19 a pandemic in March 2020. Meanwhile, the confirmed number of cases around the globe has been reported as 504,079,039, with 6,204,155 fatalities as of April 20, 2022 (https://covid19.who.int). However, Pakistan is not among the nations with the uppermost number of COVID-19 cases and fatalities. The initial case of COVID-19 was identified in Pakistan on February 25, 2020. Up to April 20, 2022, 1,527,411 COVID cases had been reported, with 30,364 fatalities (https://covid19.who.int/region/emro/country/pk).

Coronavirus pneumonia (COVID-19) is a worldwide health emergency because of its quick transmission and high death rate [39]. The clinical and physiological characteristics of SARS-CoV-2, as well as diagnostic approaches, have been studied all over the world [40]. During this pandemic, scientists and physicians face a global challenge in patient care and suitable treatment techniques, including creating an effective vaccine. Different diagnostic indicators have played a significant role in diagnosing and controlling the status of SARS-CoV-2 patients [41]. C-reactive protein (CRP) levels can be used as a biomarker to help diagnose pneumonia early, and individuals with severe lung infections have increased CRP levels [42]. Patients with COVID-19 have higher serum C-reactive protein (CRP) levels, which are used to help classify, diagnose, and make a prognosis of the disease [43]. This analysis is aimed at investigating the relationship between the length of hospital stay and CRP level, gender, age, diabetes, patient discharge status, and other comorbidities with permission of hospital authorities and consent of patient's privacy. The data was gathered from Isolation Hospital and Infectious Treatment Center (IHITC) in Islamabad from July 2021 to 30 September 2021. A total of 275 patients agreed to join in the study between July and September. All the patients admitted they belonged to Rawalpindi and Islamabad regions. We extracted information for each individual, including age, gender, diabetic status, comorbidities, length of hospital stay, CRP level, and patient discharge status.  Figure 4 illustrates the correlation graph of considered variables; this indicates the positive correlation between the hospital stay and CRP level with correlation equals 0.2 and negative correlation with other comorbidities with -0.1. However, patients' survival and age are positively associated with hospital stay with a correlation equal 0.2 and 0.1, respectively.  Figure 5 illustrates the box plot of the hospital stay. It indicates that the minimum length of hospital stay equals 1 and maximum 41, as the hospital stay is the dependent variable and contains an outlier, as shown in Figure 5. Furthermore, the residual plot of linear regression presented in Figure 6 confirms outliers in model residuals. For the out-of-sample forecast, we randomly train the model on 90% of observations (233) and validate 10% of observations (26) [23, 44, 45].

After the confirmation of outlier in the data set, the estimated model with the IIS method is defined

(13) $$\begin{array}{c} \text{Hospital stay}=\beta_{0}+\beta_{1}\text{gender}+\beta_{2}\text{age}+\beta_{3}\text{diabetes}+\beta_{4}\text{CRP}+\beta_{5}\text{survival}+\beta_{6}\text{other comorbidities}+\overset{233}{\underset{i=1}{\sum }}\gamma_{i}I_{i}+\varepsilon_{i}. \end{array}$$

Table 4 indicates that SCAD and MCP perform similarly in covariate selection, as gender, CRP level, and other comorbidities are significant variables which increase the length of hospital stay. However, SCAD selected 28 outliers, and MCP selected 31 slightly higher than SCAD.

The real data analysis confirms that the LASSO estimates more covariates and outliers than other regularization techniques, aligned with our simulation findings. LASSO selects four more than covariates selected via SCAD and MCP. Autometrics with a 5% significance chooses two covariates and 14 outliers. AdaLASSO and Autometrics with a 1% significance do not select any covariate, only retain outliers. Overall, real data analysis indicates that gender, CRP level, and other comorbidities are significant covariates. These indicator dummies can be interpreted as an observed heterogeneity of individuals, which prolonged hospital stay length. We report the RMSE of regularization techniques in Figure 7.

The above figure indicates that SCAD and MCP outperform out-of-sample RMSE compared to all other considered techniques. As expected, the LASSO selected more indicator dummies and retained higher RMSE than SCAD and MCP. With 0.01 (level of significance), Autometrics holds the highest RMSE compared to all other techniques because it dropped relevant covariate simulation finding aligned with existing studies of [20, 23]. Autometrics with tight significance levels omits relevant variables due to this RMSE increase (as observed from the simulation graph and table). In contrast, with a nominal significance level (0.05), Autometrics possesses higher RMSE than regularization techniques.

## 5. Conclusion

In cross-sectional data analysis, outlier occurred most frequently than the time series analysis, although outlier detection is a quick operation in healthcare and medical data, which is a significant cause of concern. Overall analysis indicates that regularization techniques perform more significantly than Autometrics in out-of-sample forecasting and covariate selection in simulation and real data analysis. However, the IIS method estimated via SCAD and MCP compromises promising covariate selection and forecasting results among regularization techniques. Regularization techniques with 20% and 4 SD outliers possess a higher average gauge than 20% and 6 SD. Conversely, 5% and 4 SD outlier's regularization technique possesses a higher average gauge than 5% and 4 SD outliers. Overall, with 4 SD outliers, the out-of-sample RMSE is optimal than 6 SD.

On the contrary, the LASSO estimates more outliers and covariates in simulation experiments and real data analysis than other regularization techniques. The real data analysis confirms the simulation findings, as the SCAD and MCP possess a minimum out-of-sample RMSE than Autometrics and LASSO. The real data analysis indicates that SCAD and MCP select three covariates, gender, CRP level, and other comorbidities, and possess the least RMSE. The real result is aligned with simulation findings as SCAD and MCP retain the highest potency and least RMSE compared to Autometrics. In contrast, LASSO possesses the highest gauge in simulation study compared to all considered techniques; the finding is aligned with real analysis as it retained the highest outliers. The concept of the IS method for outlier detection in the cross-sectional analysis would help to preserve unobserved heterogeneity in cross-sectional analysis, which simultaneously declines the RMSE of the estimated model. Our study proves that the IIS method for outlier detection and covariate selection estimated via SCAD and MCP gives more precise results than Autometrics in orthogonal covariates and outlier presences.

## Figures and Tables

**Figure 1:** Average RMSE with less than 5% outliers.

**Figure 2:** Average RMSE with 10% outliers.

**Figure 3:** Average RMSE with 20% outliers.

**Figure 4:** Correlation graph.

**Figure 5:** Box plot of hospital stay.

**Figure 6:** Residual box plot of linear regression.

**Figure 7:** Out-of-sample RMSE of real data analysis.

**Table 1:** Regularization penalties.

Method	Penalty function
LASSO	$P\left(.\right)=\overset{k}{\underset{j=1}{\sum }}p_{\lambda_{j}}\left(\left|\gamma_{j}\right|\right)$
AdaLASSO	$P\left(.\right)=\lambda \overset{k}{\underset{j=1}{\sum }}{\hat{w}}_{j}{\left|\gamma_{j}\right|}_{1}$
SCAD	$P\left(.\right)=\overset{k}{\underset{j=1}{\sum }}p_{j}\left(\left|\gamma_{j}\right|;\lambda ;\alpha \right)$
MCP	$P\left(.\right)=\overset{k}{\underset{j=1}{\sum }}p_{j}\left(\left|\gamma_{j}\right|;\lambda ;\alpha \right)$

*p*_*λ*_*j*__(.) is a function denoted as penalty function, and *λ*_*j*_ is the function parameter.

**Table 2:** Simulated results with different percentages of outliers with 6 SD.

20% outliers		
	Gauge	Potency
SCAD	0.222	0.367
MCP	0.222	0.367
LASSO	0.611	0.767
AdaLASSO	0.333	0.433
Auto(0.05)	0.011	0.100
Auto(0.01)	0.011	0.100
10% outliers		
SCAD	0.100	0.500
MCP	0.140	0.550
LASSO	0.650	0.850
AdaLASSO	0.220	0.600
Auto(0.05)	0.010	0.200
Auto(0.01)	0.000	0.200
5% outliers		
SCAD	0.048	0.600
MCP	0.048	0.600
LASSO	0.591	0.933
AdaLASSO	0.124	0.667
Auto(0.05)	0.000	0.534
Auto(0.01)	0.000	0.534

**Table 3:** Simulated results with different percentages of outliers with 4 SD.

20% outliers		
	Gauge	Potency
SCAD	0.222	1.000
MCP	0.144	1.000
LASSO	0.611	0.967
AdaLASSO	0.189	0.933
Auto(0.05)	0.000	0.367
Auto(0.01)	0.011	0.367
10% outliers		
SCAD	0.230	0.600
MCP	0.150	0.550
LASSO	0.650	0.850
AdaLASSO	0.360	0.700
Auto(0.05)	0.000	0.500
Auto(0.01)	0.000	0.500
5% outliers		
SCAD	0.114	0.667
MCP	0.095	0.667
LASSO	0.657	0.867
AdaLASSO	0.352	0.667
Auto(0.05)	0.000	0.667
Auto(0.01)	0.000	0.667

**Table 4:** Real data analysis with covariate selection and number of selected outliers.

SCAD number of selected outliers (28)				
Variable	Gender	CRP level	Other comorbidities	
Coefficient	0.24463	0.00083	0.20533	
MCP number of selected outliers (31)				
Variable	Gender	CRP level	Other comorbidities	
Coefficient	0.22493	0.0004	0.2585	
LASSO number of selected outliers (204)				
Variable	Age	Gender	CRP level	Other comorbidities
Coefficient	0.00225	0.55747	0.00282	1.3966
Auto(0.05) number of selected outliers (14)				
Variable	CRP level	Other comorbidities		
Coefficient	0.00766	0.9653		

## Data Availability

Data can be provided on request.
